# Efficient Automated Disease Diagnosis Using Machine Learning Models

**DOI:** 10.1155/2021/9983652

**Published:** 2021-05-04

**Authors:** Naresh Kumar, Nripendra Narayan Das, Deepali Gupta, Kamali Gupta, Jatin Bindra

**Affiliations:** ^1^Department of Computer Science & Engineering, Maharaja Surajmal Institute of Technology, C-4, Janakpuri, New Delhi 110058, India; ^2^Department of Information Technology, School of Computing and Information Technology, Manipal University Jaipur, Jaipur, Rajasthan 303007, India; ^3^Chitkara University Institute of Engineering and Technology, Chitkara University, Rajpura, Punjab, India

## Abstract

Recently, many researchers have designed various automated diagnosis models using various supervised learning models. An early diagnosis of disease may control the death rate due to these diseases. In this paper, an efficient automated disease diagnosis model is designed using the machine learning models. In this paper, we have selected three critical diseases such as coronavirus, heart disease, and diabetes. In the proposed model, the data are entered into an android app, the analysis is then performed in a real-time database using a pretrained machine learning model which was trained on the same dataset and deployed in firebase, and finally, the disease detection result is shown in the android app. Logistic regression is used to carry out computation for prediction. Early detection can help in identifying the risk of coronavirus, heart disease, and diabetes. Comparative analysis indicates that the proposed model can help doctors to give timely medications for treatment.

## 1. Introduction

Machine learning is used in various areas like education and healthcare. With the advancement of technology, the better computing power and availability of datasets on open-source repositories have further increased the use of machine learning. Machine learning is used in healthcare in vast areas. The healthcare sector produces large amounts of data in terms of images, patient data, and so on that helps to identify patterns and make predictions. Machine learning is used in healthcare to solve various problems [1–3]. Heart disease is based on the individual, and the extent of heart disease can vary from person to person [4]. Thus, making a machine learning model, training it on the dataset, and entering individual patient details can help in prediction. The prediction result will be according to the data entered and hence will be specific to that individual. Type-2 diabetes is a disease that can be prevented by control of weight, lifestyle, and so on [5]. Coronavirus is a disease that has no clearly defined treatment. The coronavirus 2019 (COVID-19) originated from China. There are different treatments [6] that are going on for it but there are no clearly defined steps for treatment.

Artificial intelligence (AI) aims to mimic human cognitive functions. It is bringing a paradigm shift to healthcare, powered by the increasing availability of healthcare data and rapid progress of analytics techniques [1]. Recently, many models have been developed for automated diagnosis of various diseases such as cancer, COVID-19, and diabetes [2]. Recently, many researchers have started using machine learning models for real-time diagnosis of disease by developing mobile apps [3]. Even some mobile apps have been developed which can predict the risk of certain disease and recommend the diagnosis to the given person based upon the respective health conditions [4]. However, efficient early stage diagnosis is still defined as an ill-posed problem [5]. Recently, many researchers have started using deep-learning models to obtain significantly better performance as compared with the machine learning models [6, 7].

In this study, the machine learning models are applied to the coronavirus, heart disease, and diabetes dataset to predict the risk of these diseases in an individual. An end-to-end process is used where people must enter their details in the mobile application and submit the data. The real-time processing takes place, and the risk is predicted within a few seconds. The mobile application that is used as a real-time database on the cloud is the firebase database. The trained parameters of the model are stored in the database, and prediction is done in real-time. Further, the user is also notified of the accuracy of the model. Apart from this, the news article from trusted sources is also shared in the app in real-time. The source of the news is also mentioned in the app.

The main contributions are as follows:

- An efficient automated disease diagnosis model is designed using the machine learning models.
- Three critical diseases are selected such as coronavirus, heart disease, and diabetes.
- In the proposed model, the data are entered into an android app, the analysis is then performed in a real-time database using a pretrained machine learning model which was trained on the same dataset and deployed in firebase, and finally, the disease detection result is shown in the android app.
- Logistic regression is used to carry out computation for prediction.

The remaining paper is summarized as follows.  Section 2 presents related work.  Section 3 presents the research methodology.  Section 4 discusses the experimental results and analysis.  Section 5 concludes the paper.

## 2. Related Work

Machine learning is used widely in today's world because of increasing computation power and the availability of large datasets on open-source tools. Quality of transmission (QoT) can give some insights into the model. An attempt has been made to monitor the QoT to determine the physical condition of the model [7]. In another study, an attempt has been made to use ML in intrusion detection systems [8–10]. Song et al. [11] proposed a modified optimization method for the extreme learning machine. In another study, a supervised deep-learning technique is used to diagnose faults in the induction machine system [12]. ML is also used in demodulation methods [13] for visible light communication systems. In wireless networking, resource management is another problem where ML was applied to obtain optimal performance [14].

In another study, an algorithm is proposed to achieve local updates and global updates [15] which is critical for the learning process. ML is also used to solve wireless network problems. Chen et al. [16] represented how artificial neural networks can be used to solve various problems in the wireless network. Nawaz et al. [17] gave a detailed study of how different models are used in 5G technology. In another study [18], detailed research is presented on how neuromorphic photonics systems are used in solving ML-based problems. An attempt has been made to detect falls and daily activity using artificial neural networks [19]. An attempt has been even made for the diagnosis of ML models [20]. ML is also used to detect malware in android software [21]. Tang et al. [22] provided insights for the use of ML in vehicular 6G networks. ML is also used to determine flight delay [23]. In another attempt, ML is used to determine the protein dynamics [24]. In another study, the use of AI in wireless communication [25] is done and the new research area developed is called edge learning.

The use of machine learning models in healthcare has increased. The ability of machine learning models to bring out the meaning from data and to prediction is used for early prediction of diseases. Machine learning is used in heart disease problems to bring out solutions to complex problems. For instance, some data mining techniques are applied to heart disease data [26] to determine patterns and help in the prediction of heart disease. In another study [27], a hybrid of machine learning models is proposed for the diagnosis of heart disease. Khourdifi and Bahaj [28] used different machine learning models for heart disease prediction and applied various optimizations which include particle swarm optimization (PSO) combined with ant colony optimization (ACO). In a study, [29] ensemble technique is used for the prediction of heart disease. Their research showed that the ensemble technique increased the accuracy of weak classifiers. Several studies have tried to link heart disease with coronavirus to determine if there is any relation among them [30–35]. There are several attempts made to determine heart disease and prevent it before it causes serious harm [36–40].

The machine learning models are also used for coronavirus disease to solve problems in the medical domain using data. For instance, machine learning techniques and mathematical models are used [41] to determine the number of infected people and the probable time when coronavirus will be over in China. In a study conducted by Bullock [42], various applications, tools, and datasets are explored which bring in the artificial intelligence used against coronavirus. The role of artificial intelligence and machine learning to fight coronavirus is necessary as it will help in the early prediction of coronavirus [43]. In the coronavirus situation, it is necessary to characterize the propagation of information on social media [44]. The patients who have hypertension and diabetes [45] or have old age [46] are at higher risk of coronavirus [47]. An attempt has been made to determine the relation between coronavirus and diabetes [48–51].

Diabetes has been in society for a very long time. Diabetes is further dependent on an individual's body, diet, and way of living [5]. Machine learning models are used in diabetes problems to bring out solutions and to enable early prediction using machine learning models. For instance, Alghamdi et al. [52] developed an ensemble-based model for predicting incident diabetes. The database used in the research has 32,555 patients. In another study, prediabetes is predicted using machine learning models on the Korean population [53]. Sneha and Gangil [54] analyzed the dataset for selecting the optimal features for the early prediction of diabetes. Zou et al. [55] used a dataset of Luzhou, China, to predict and diagnose diabetes. An attempt has been made to identify diabetes in developing countries [56]. Diabetes is more in older people than in younger generations, so an attempt has been made to list the clinical procedure for handling diabetes in older adults [57].  Table 1 presents the comparative analysis among the existing techniques.

## 3. Methodology

The objective of the methodology is to predict the risk of having coronavirus, heart disease, and diabetes in an individual based on answering a few questions using machine learning models in an end-to-end process. The research is carried on a system with the following system configurations and software: Python 3 and Java 10.0.2 software are used and implemented using Jupyter Notebook 5.5.0 and Android Studio 3.1.0, respectively, on Intel(R) Core(TM) i3-2310M CPU @2.10 GHz with 8 GB RAM.

A block diagram of the basic steps adopted for each machine learning model is shown in Figure 1. First, data cleaning is performed to convert the raw data into a usable form. After data cleaning, data analysis is done to determine the importance of features. In data analysis, the features are identified, and the data are converted into a form on which machine learning models can be applied. These steps are used for each of the model predictions: (a) COVID-19, (b) heart disease, and (c) diabetes.

### 3.1. COVID-19

The data of COVID-19 collected from [18, 58] include many features which are represented in Table 2. The dataset is raw and cannot be used directly. The total data points of the dataset are 13174. However, most of the data points have missing values. For instance, 11825 age value, 12681 symptoms value, 12416 travel history location, and so on are missing. The relevant features selected include age, sex, symptoms, country, and travel_history_location. These values are essential to carry out predictions. However, due to missing values, many data points are dropped. After removing the null values, the dataset consists of 260 rows. A view of the dataset after cleaning is shown in Table 3.

After data cleaning, data analysis is performed. After cleaning the dataset, there are 260 rows. The country columns include following countries: “China,” “France,” “Japan,” “Malaysia,” “Nepal,” “Singapore,” “South Korea,” “Thailand,” “United States,” “Cambodia,” “Vietnam,” “Philippines,” “Italy,” “Lebanon,” “Spain,” “Lithuania.” These countries were segregated into two separate groups: the first one with countries having more than 10,000 cases and the second one with less than 10,000 cases. The data points in the first group are marked by 1 in the country column, and data points in the second group are marked by 0 for the country column. Data points that had no travel history were marked by 0, and the rest were marked by 1. For the sex column, the male was marked by 0 and the female was marked by 1. The complete dataset of COVID-19 consists of only the details of patients tested positive. To apply machine learning models, the dataset must have negative cases also; otherwise, the model will predict all cases positively based on learning. For this reason, 80 new rows were added with a negative result. Here, 0 entry in the output column corresponds to a negative result. The age and sex of these 80 data points were the same as the first 80 data points of the dataset. The columns-symptoms, country, and travel_history_location were made to cover all possible 8 cases. 10 rows correspond to each case. After completion of the dataset, a heat map was drawn to determine the impact of each feature on the prediction of output.

In Figure 2, analyzing the heatmap, it can be seen that symptoms and travel history location have a huge positive impact on having the COVID-19.

### 3.2. Heart Disease

The heart disease dataset [19, 59] has features shown in Table 4. The dataset has 70,000 data points. Out of the features listed in the table, the features used include “age,” “gender,” “height,” “weight,” “cholesterol,” “gluc,” “smoke,” “alco,” “ap_hi,” and “ap_lo.” There were some outliers. The value of systolic blood pressure above 200 and the value of diastolic pressure above 150 are referred to as outliers here. A snapshot of the dataset is shown in Figure 3.

For analysis of features, a heat map was drawn. According to the heat map (see Figure 3), the most important features in determining heart disease include systolic and diastolic blood pressure, cholesterol, and age (see Table 5).

### 3.3. Diabetes

The dataset collected from [20, 60] has the features as shown in Table 6. The dataset has 768 data points. Out of all the listed features in Table 3, the features used include “pregnancies,” “blood pressure,” “BMI,” and “age.” The aim of the research is not only to build a theoretical model of prediction by using artificial intelligence but to make it practically possible to use the models in the real-time application without many restrictions. The features including skin thickness and diabetes pedigree function are not possible for a normal person to determine at home. For this reason, only those features are taken which are possible for predicting. For instance, diabetes pedigree function is a complex function [61] calculated by using various factors including parents, siblings, half aunt, and half-uncle. A view of the dataset is shown in Table 7.

A heat map was drawn to determine the importance of features. According to the heat map, pregnancies, glucose, BMI, and age have the highest impact (greater than 0.2) on predicting diabetes (see Figure 4). Out of this, glucose is not considered for making the model useful for practical use (see Table 7).

After cleaning and analyzing all the datasets, machine learning models were applied. The logistic regression model is used for all the datasets. To make the prediction, the coefficients and intercept of all the three logistic regression models are stored in a firebase real-time database. Since coefficients and intercept are in the firebase real-time database, any updation in the coefficients can be reflected in real-time in the application. This allows us further to tweak the parameters as the dataset grows and training improves. To make it useful for practical use, an android application is developed. Using the android application, the prediction can be made in real-time by answering a few questions. To further make the application useful, all the latest news and trends of COVID-19, diabetes, and heart disease are shown in the app that can be updated in real-time.

## 4. Results and Discussion

Figure 5 shows an example of prediction in the android app. The screenshots used in Figure 5 are taken from the android app in production, which is named disease prediction using artificial intelligence (DPAI). The user can choose from various options to predict diseases or look at news/trends of diseases from the main navigation menu as shown in Step 1. The user must enter some details which are features fed to the model for prediction. For prediction, the value of various coefficients and intercept is fetched from the firebase database in real-time, and calculation is performed to give the output. Along with the output, the accuracy of the model is also displayed to users for more transparency.

In this paper, we have used 65% dataset for training process, 10% for cross-validation, and 25% for testing purpose. Figures 6–8 show the accuracy analysis of the proposed and the existing machine learning models by considering diabetes, heart disease, and COVID-19 binary datasets. These figures clearly show that the proposed model outperforms the existing models by 1.2746%. Figures 9–11 demonstrate the F-measure analysis of the proposed and the existing machine learning models by considering diabetes, heart disease, and COVID-19 binary datasets. These figures clearly show that the proposed model outperforms the existing models by 1.3926%.

From the comparative analysis, it is found that among the existing models, the proposed model outperforms the competitive models in terms of various performance measures. Also, the proposed model provides consistently good performance with lesser degree of uncertainty, especially compared with LR, J48, KNN, ANN, RF, GB, and ANFIS.

## 5. Conclusion

This study provides insights into using the machine learning models to predict the risk of COVID-19, heart disease, and diabetes in an individual based on answering a few questions related to various factors like travel history, age, gender, and blood pressure. Logistic regression is used for prediction. Extensive experimental results reveal that the proposed model outperforms the competitive machine learning models in terms of accuracy and F-measure by 1.4765% and 1.2782, respectively, for COVID-19 dataset. The proposed model outperforms the competitive machine learning models in terms of accuracy and F-measure by 1.8274% and 1.7264, respectively, for diabetes dataset. Also, the proposed model outperforms the competitive machine learning models in terms of accuracy and F-measure by 1.7362% and 1.3821, respectively, for heart disease dataset.

The findings in this research can be helpful in the early screening of potential COVID-19, diabetes, and heart disease patients. It can be helpful in the sense that the first screening can be performed at the comfort of home. If a high risk of disease is predicted in a patient, then it can be followed by clinical trials for confirmation. In the near future, one may apply the proposed model to some other applications such as handwritten recognition [62], image filtering [63], cancer classification [64], and medical image segmentation [65] and additionally may use various meta-heuristic techniques [66] to tune the initial parameters of the proposed machine learning models.

## Figures and Tables

**Figure 1:** Diagrammatic flow of the proposed methdology.

**Figure 2:** Heatmap of COVID-19 dataset.

**Figure 3:** Heat map of heart disease dataset.

**Figure 4:** Heatmap of diabetes dataset.

**Figure 5:** Prediction steps.

**Figure 6:** Accuracy analysis on diabetes dataset.

**Figure 7:** Accuracy analysis on COVID-19 dataset.

**Figure 8:** Accuracy analysis on heart disease dataset.

**Figure 9:** F-measure analysis on diabetes dataset.

**Figure 10:** F-measure analysis on COVID-19 dataset.

**Figure 11:** F-measure analysis on heart disease dataset.

**Table 1:** Comparative analysis of the existing techniques.

Ref.	Year	Model	Features	Application
[2]	2019	Machine learning models	Used general linear model (GLM) regression, support vector machines (SVMs) with a radial basis function kernel, and single-layer artificial neural networks	Medicine
[3]	2019	Artificial intelligence in healthcare	AI can perform healthcare tasks as well or better than humans, implementation factors will prevent large-scale automation of healthcare professional jobs for a considerable period	Healthcare
[4]	2016	—	In addition to individual CVD risk factors, Framingham and systematic coronary risk evaluation (SCORE) algorithms were used to assess the absolute risk of a CVD	Open heart
[6]	2020	DenseNet201	A DenseNet201-based deep transfer learning (DTL) is proposed to classify the patients as COVID infected or not, i.e., COVID-19 (+) or COVID (−)	COVID-19
[8]	2019	Deep learning	A Comprehensive analysis was presented on the use of machine and deep learning for IDS systems in wireless sensor networks (WSNs)	Wireless networks
[26]	2016	Data mining technique	Decision tree shows better results as compared with J48, logistic model tree algorithm, and random forest	Heart disease
[27]	2016	Heart disease	The features reduction has an impact on classifiers performance in terms of accuracy and execution time of classifiers	Medical
[28]	2019	Machine learning	Artificial neural network optimized by particle swarm optimization (PSO) combined with ant colony optimization (ACO) approaches	Heart disease
[29]	2019	Ensemble classification techniques	The ensemble technique can be applied for improving prediction accuracy in heart disease	Medicine
[30]	2020	Deep transfer learning	Used to detect and diagnose COVID-19. Chest X-rays is preferred over CT scan	COVID-19
[32]	2020	Deep convolutional neural networks	Computed tomography (CT) scans to diagnose pneumonia, lung inflammation, abscesses, and enlarged lymph nodes. Since COVID-19 attacks the epithelial cells that line our respiratory tract, therefore, X-ray images are utilized	COVID-19

**Table 2:** Features of the dataset.

	Age	Sex	Symptoms	Country	Travel _history location	Outcome
0	42	Female	Fever	China	Wuhan	1
1	59	Female	Fever	China	Wuhan	1
2	38	Female	Cough	China	Wuhan	1
3	45	Male	Fever	China	Wuhan	1
4	33	Female	Fever	China	Wuhan	1

**Table 3:** Features in COVID-19 dataset.

ID	date_admission_hospital	Sequence available
Age	Date confirmation	Outcome
Sex	Symptoms	date_death_or_discharge
City	lives_in_Wuhan	notes_for_discussion
Province	travel_history_dates	Location
Country	travel_history_location	admin3
Wuhan(0)_not Wuhan(1)	reported_market_exposure	admin2
Latitude	Additional information	admin1
Longitude	chronic_disease_binary	Country new
geo_resolution	Chronic disease	admin_id
date_onset_symptoms	Source	data_moderator_initials

**Table 4:** Heart disease dataset.

	Id	Age	Gender	Height	Weight	Ap_lo	Cholesterol	Gluc	Smoke	Alco	Active	Cardio
0	0	18393	2	168	62.0	110	80	1	1	0	1	0
1	1	20228	1	156	85.0	140	90	3	1	0	1	1
2	2	18857	1	165	64.0	130	70	3	1	0	0	1
3	3	17623	2	169	82.0	150	100	1	1	0	1	1
4	4	17474	1	158	58.0	100	60	1	1	0	0	0

**Table 5:** Features in heart disease dataset.

Feature	Description
Age	Days-integer
Height	Height in cm-integer
Weight	Weight in kg-float
Gender	Categorical code (1-women, 2-men)
Systolic blood pressure	Integer
Diastolic blood pressure	Integer
Cholesterol	1: normal, 2: above normal, 3: well above normal
Glucose	1: normal, 2: above normal, 3: well above normal
Smoking	Binary
Alcohol intake	Binary
Physical activity	Binary
Presence or absence of cardiovascular disease	Binary

**Table 6:** Features in diabetes dataset.

Features	Description
Pregnancies	Number of times pregnant
Glucose	Plasma glucose concentration 2 hours in an oral glucose tolerance test
Blood pressure	Diastolic blood pressure (mm Hg)
Skin thickness	Triceps skin fold thickness (mm)
Insulin	2-hour serum insulin (mu U/ml)
BMI	Body mass index (weight in kg/(height in m)^2)
Diabetes pedigree function	Diabetes pedigree function
Age	Age (years)
Outcome	Class variable (0 or 1)

**Table 7:** Diabetes dataset.

	Pregnancies	Glucose	Blood pressure	Skin thickness	Insulin	BMI	Diabetes pedigree function	Age	Outcome
0	6	148	72	35	0	33.6	0.63	50	1
1	1	85	66	29	0	26.6	0.35	31	0
2	8	183	64	0	0	23.3	0.67	32	1
3	1	89	66	23	94	28.1	0.17	21	0
4	0	137	40	35	168	43.1	2.29	33	1

## Data Availability

The data used to support the findings of this study are available from the corresponding author upon request.
